# Labor Culture and Ecological Environment: The Renewing Path of the Nurturing Concept of “Nurturing Talents for the Country” in Labor Education

**DOI:** 10.1155/2022/6563526

**Published:** 2022-09-29

**Authors:** Wei Hu, Kun Ma

**Affiliations:** ^1^Chongqing Creation Vocational College Personnel Department, Yongchuan, Chongqing 402160, China; ^2^Chongqing Creation Vocational College School (Youth) League Committee, Yongchuan, Chongqing 402160, China

## Abstract

It is the responsibility of colleges and universities to nurture talents for the country. In the final analysis, the purpose of teaching, scientific research, and social services in colleges and universities is to educate people. The study of labor education, in the face of the important historical opportunity of transformation, is a theoretical representation of labor education and its value choice. The answer to this question can help us clarify the meaning of labor education and improve the scientific and systematic practice of labor education. Labor education in colleges and universities has an important and extensive value significance for cultivating contemporary college students, which can not only inspire students to study hard in science and culture, master their skills, and grow their talents but also guide them to firm ideals and beliefs, exercise good character, and cultivate the emotional experience of labor so that contemporary college students can integrate the pursuit of life values with the great cause of national prosperity and national rejuvenation and integrate the beautiful vision of personal ambition and family happiness with the good cause of collective, social, and national interests. This paper is based on the background of the times. Therefore, this paper studies the labor culture and ecological environment from the background of the times: the path of renewing the concept of “cultivating talents for the nation” in labor education. It also gives a profound discussion on labor education in high schools and finally puts forward relevant suggestions for the problems.

## 1. Introduction

The study of labor education is a theoretical representation of labor education and its own value choice in the face of the important historical opportunity of the transformation of the times. They can combine their personal ambition and family happiness with the community of development and destiny, which integrates collective, social, and national interests [1]. It is of theoretical and practical significance to strengthen the research on the innovation of labor education methods in colleges and universities in the new era. The effect of labor education is influenced by the purpose, content, subject and object, environment, carrier, and other aspects. Although labor education is characterized as “education,” its implementation path is not only based on the school curriculum but also emphasizes the practice of labor education. China has a long history of providing labor education courses [2]. At present, although the relevant opinions issued by the Party Central Committee and the implementation of the relevant planning outline have made important arrangements and top-level design for labor education in colleges and universities, there is still a need for in-depth discussion on the innovation of labor education in colleges and universities. In terms of labor education theory research, the basic connotation, important significance, and institutional mechanism of innovation of labor education methods in colleges and universities in the new era need to be explored in depth [3].

## 2. Research Background

General Secretary Xi Jinping has made a profound discussion on labor education. The discourse explains the important status of labor education, which is not only a way for the comprehensive development of youth but also takes up the historical responsibility of working together with moral, intellectual, physical, and aesthetic education to cultivate qualified newcomers of the times [4]. Colleges and universities should assume the main responsibility of organizing and guiding the development of students' ideological education in order to promote the reform and innovative development of labor education, cultivate the labor sentiment of contemporary college students, and make the cause of national rejuvenation obtain the dedicated participation of a batch of qualified talents [5].

It is the responsibility of colleges and universities to nurture talents for the country. In the final analysis, the purpose of teaching and conducting scientific research and social services in colleges and universities is to nurture people. Since the 18th National Congress, Xi Jinping has repeatedly requested to make efforts in labor education, so as to strengthen the cultivation of labor values and make college students realize the truth that “labor is the most honorable, noble, and beautiful.” To strengthen the moral cultivation, we must cultivate the excellent labor quality of college students and teach them to struggle hard, work honestly, innovate, and dedicate; to increase knowledge and insight, we must strengthen the cultivation of scientific labor skills and labor practice training, so as to move forward in the right direction of seeking the truth, understanding the truth and understanding things; to cultivate the spirit of struggle, we must strengthen social labor practice, further. To make efforts in cultivating the spirit of struggle, we should strengthen social labor practice, further promote the integration of industry and education, and solidly promote college students to truly grasp hard work and take up struggle in the social melting pot; to make efforts in enhancing comprehensive quality, we should give full play to the comprehensive educational value that labor naturally possesses and organically incorporate labor education into the teaching system of comprehensive development [6].

It is conducive to promote the practical development of labor education way innovation in colleges and universities in the new era. The practice of labor education in colleges and universities in the new era is still at the initial stage, and there are many difficult problems that need to be solved. Innovation of labor education methods to the effectiveness of labor education. “What contents should be taught in school education and what ways should be adopted to impart these contents to students, so as to stimulate students' interest in knowledge to reach educational goals.” The innovation of labor education methods can solve the problem of how to teach labor education and how to attract students, as a way to enhance the modernity and scientificity of labor education methods [7].

## 3. Materials and Methods

### 3.1. Basic Theories

#### 3.1.1. Labor Education

The General Secretary's important discourse on labor education is of great significance in improving the concept of five education and three comprehensive education, while this discourse is an important part of the development and improvement of the Marxist labor education ideology under the new stage and new conditions, which is of great significance in helping students to establish good moral character and has important theoretical significance for the long-term development of China's education [8], as shown in Figure 1.

Labor education is a very important part of it, and it is important for promoting moral, intellectual, physical, and aesthetic education, and Xi Jinping's important discussion on labor education is important for promoting the implementation of the “five education” concept of comprehensive development [9].

To cultivate morality through labor, the formation of a person's moral character is mainly influenced by his acquired education and experience. In the ancient times, “Heaven is healthy, and a gentleman is self-improving.” In the ancient times, “Heaven is healthy, and a gentleman is strong by self-improvement,” emphasizing the formation of moral character through diligence and hard work. “Therefore, if Heaven will give a great task to a man, he must first suffer his heart and mind and labor his muscles and bones.” It can be seen that labor has always been closely related to character building, and General Secretary Xi Jinping called for the promotion of labor education to promote people to establish the good virtues of perseverance, hardship, and hard work in serious and practical labor and in ordinary daily work, to enhance the sense of social responsibility and morality of workers, and to promote moral construction [10].

Increasing wisdom with labor, the composition of people's knowledge mainly includes direct experience and indirect experience, both of which have the same status and importance. Indirect experience is the experience of the previous people; the experience that has been summarized and organized by others to form literal theories and conclusions. Direct experience is the experience that individuals gain through their own actual feelings and experiences in practical activities and behaviors. Indirect experience gives people theoretical guidance and basic direction and is the absorption of valuable human knowledge, while direct experience is the experience people accumulate directly in real life, which has the characteristics of more intuitive, more visual, and more vivid. In order to grow into a fully developed and socially progressive person, it is far from enough to learn knowledge from books and to learn only from the words in books, but it is necessary to accumulate enough direct experience to obtain real growth. Labor activity is an important practical activity for human beings to gain direct experience, in which people increase their technical skills to cope with different situations and problems and constantly sum up the methods to solve various problems.

Strengthening the body with labor. Mao Zedong pointed out the importance of strong national body and strong will for national development and national rejuvenation. A strong body is the basis and prerequisite for people to do all work well, and the body is the capital of revolution. The physical quality of young students is not only about their personal future and development but also about the overall quality of the nation, which is an important symbol of the development and prosperity of a country and the happiness of its people. Through labor education, organization of labor activities, and labor courses, we can help students get exercise in labor activities, strengthen their physical strength, and create conditions for their work development.

Educating beauty through labor, the beauty of a person includes both inner and outer beauty. On the one hand, carrying out labor education and guiding students to participate in labor activities can strengthen students' physique, increase students' vitality, help students maintain a balanced and slim physique, and promote students to face life with a high and upward appearance, thus increasing students' external beauty. On the other hand, by organizing students' labor and participating in practical activities, it can help students forge a good character of hard work, diligence, and courage, cultivate the labor spirit of dedication and excellence, lay a good foundation for students to shine in their future positions, help students realize their self-worth through labor, enhance their sense of gain, satisfaction, and achievement in life, enhance their self-confidence, and show their youthful power. It also helps students to enrich their inner beauty.

Xi Jinping's important statement on labor education promotes the scientific education concept of “three-wide education.” The requirement of “three-whole education” is to educate the whole person, the whole process, and the whole range of people. The implementation of labor education is essentially the implementation of the concept of “three-wide education.” First of all, the purpose of integrating labor education into the whole process of human resource training, from elementary school to university, is to integrate labor into all processes of education and teaching, which reflects the idea of nurturing people in the whole process. In the process of labor education, we follow the objective laws of education and progress step by step, helping students to establish correct labor concepts by promoting correct labor values, enriching labor knowledge and improving labor quality by establishing labor courses, improving labor skills by organizing labor activities, gradually advancing from labor concepts to labor knowledge to labor skills, and integrating labor education in all aspects and processes of education and teaching. Secondly, we advocate that labor education is not only the responsibility of schools but also requires the cooperation of families and the support of society. Labor education is not only the responsibility of schools but also the responsibility of families and society, and the effective promotion of labor education cannot be achieved without the joint efforts and cooperation of all three parties. By organizing students' household activities and helping their parents to solve some trivial household tasks, families foster the correct awareness of paying attention to personal health and hygiene, develop good habits of hard work, improve students' skills of independent living, and get rid of students' extreme dependence on their parents and families [11]. Schools improve students' ability to master labor knowledge and theory through labor courses and labor knowledge education, while society helps students improve their labor ability by providing them with a platform for practical and labor activities, helping them to further complete the socialization process and become high-quality talents who can adapt to the development and needs of society. It can be seen that the promotion of labor education cannot be separated from the efforts of any party in school, family, and society and requires the coordination and systematic optimization of all parties in school, family, and society, and insisting on the coordination of all parties in family, school, and society is an important embodiment and perfect development of the scientific education concept of “three comprehensive education” [12]. The five-education, three-whole concept is shown in Figure 2.

#### 3.1.2. “Nurturing Talents for the Country” Concept

“Nurturing talents for the country” is the fundamental task of talent cultivation in China. In ancient times, China advocates “cultivating oneself, preparing one's family, ruling the country, and pacifying the world,” emphasizing that the governance of political clarity and harmony should start from the internal moral cultivation of individuals. Eventually, the world will be governed [13]. Xi Jinping's emphasis on “understanding great virtue, abiding by public virtue, and being strict with private virtue” specifies the requirements and contents of moral cultivation of character in “cultivating talents for the country.” Labor is an important practical activity that sustains human survival and development, and labor morality is an important part of personal morality. Through labor education, students are helped to develop good moral character by making their own efforts to gain from simple labor activities, so as not to make any mistake about their names. The goal of “education for the nation” is implemented. Unlike the education and teaching of theoretical knowledge, labor education is a kind of practical education, which helps students learn by doing and practice by learning. Through organizing students to carry out labor practice activities, grassroots posting activities, and social volunteer activities, students can improve their level of facing challenges and overcoming difficulties, sharpen their willpower of perseverance, enhance their ability to help others and repay society, and cultivate their character of putting others before themselves and actively contributing to society. We also aim to enrich the content of the education concept of education for the country. It is not enough to cultivate students' character only from theoretical knowledge, students can have a basic idea of character, but theoretical knowledge is too abstract and lack real feeling and experience of character establishment. The students will be able to understand the spirit of hard work, courage, courageousness, and perseverance. Students are helped to integrate these good virtues into their own practice, to get rid of the stereotypical impressions and senses of establishing good virtues, and to form their own true feelings about serving others and society [14].

On the one hand, Marx and Engels followed the laws of materialistic dialectics to emphasize the need to achieve a combination of productive labor and education and to cultivate people who achieve comprehensive development in all aspects, highlighting the importance of labor for social progress as well as personal advancement [15]. On the other hand, Xi Jinping has made many visits and explorations to improve and practice Marx and Engels' thought of labor education on the basis of the current situation of China's educational development and the process of social development and has made a new judgment and positioning of the value of labor education in the era, by guiding the people to form a correct concept of labor, improving the labor literacy of the working masses, realizing the cultivation of character and forging will through labor, and improving people's intelligence through labor activities. Through labor activities, people's intellect is enlightened, their discernment is improved, their physical condition is improved, and their personality is enhanced through labor, and the Marxist concept of labor education is made practical, concrete, and enriched by incorporating labor education into the whole process of human resources training, throughout the school years from elementary school to university, and in all aspects. These important statements specify the essence of labor education and, in the process of practice, insist on following the pursuit of truth and basing on facts, build a good platform for students to grow in labor and practice, provide ways to practice labor, improve students' social life skills, and raise their labor level. Encourage students to dare to go out of their comfort zone and carry out some meaningful and valuable work in places where the development of the motherland is urgently needed, help students resist temptation in the complicated society, establish a correct outlook on life, worldview and values, and make labor education take on a new look in the new era.

#### 3.1.3. Ecological Environment Improvement Theory

Habitat is the environment suitable for human habitation. With rapid population growth, people's living conditions are deteriorating, and the problem of human settlements is of increasing concern [16]. Both developed and developing countries face the same human settlement problems: overpopulation, underfunding of basic services, inadequate housing, and deteriorating infrastructure; 40 to 50 percent of the world's population lives in slums [17].

UN-HABITAT was established in 1978 as the leading agency within the UN system for coordinating human settlement development, supporting and collaborating with governments, local authorities, nongovernmental organizations and the private sector to promote global human settlement development [18], as shown in Figure 3.

First, the majority of low-income people in all regions of the world do not have access to adequate housing and social services. In developing countries, at least 600 million urban dwellers live in poor conditions with inadequate access to drinking water, sanitation, hygiene, and waste disposal, which pose a constant threat to their lives and health. One million urban dwellers are forcibly evicted from their homes each year, bringing the number of homeless people to an estimated 100 million. Habitat assists in the development of policies, strategies, and supply systems for housing and social services. The center promotes the full and progressive realization of the right to housing through the development of appropriate housing policies with community participation and calls on governments to remove institutional and regulatory constraints that impede access to land and housing.

Second, by the year 2000, half of the world's population will be living in cities. By 2030, the urban population will be twice as large as the rural population. Rapid urbanization, concentration of urban populations in large cities, massive urbanization, and rapid expansion of megacities are among the most important changes of our time. As a result, the development of almost every country today will depend to a large extent on its ability to manage its cities. Recognizing that local authorities may be the most effective partners in building more productive, equitable, and sustainable urban areas, the center is committed to working closely with local authorities and other city administrations to implement the Habitat Agenda at the city level.

Once again, urban development related to the environment and infrastructure can provide important opportunities for sustainable development, as cities can effectively accommodate large numbers of people in a limited space. However, without proper planning and management of the environment and infrastructure, cities will become major sources of air pollution, water pollution, poor sanitation, and serious health, environmental, and economic problems caused by human activities and natural disasters. Determined to improve people's living conditions, it supports governments, local authorities, and communities in planning, implementing, and maintaining infrastructure and services in urban and rural human settlements and promotes the development of local environmental policies, especially in the areas of water supply and waste management, wastewater treatment, transportation, and energy.

Finally, through its Global Urban Observatory, the center monitors and oversees implementation at the global level through two main monitoring tools, the Best Practices Project and the Urban Indicators Project. The results of these observations are published in the State of the World's Cities Biennial Report. The center's worldwide press offices, targeted information materials, the Internet, and its two main periodicals, the Global Report on Human Settlements and the Habitat Debate, have contributed to raising awareness of the sustainable development and urban agenda for political change in favor of society as a whole, as well as economic and environmental issues in an urbanizing world [19]. The development of eco-environmental theory has evolved in three stages as shown in Figure 4.

### 3.2. Main Evaluation Methods

In this paper, an ant colony algorithm is used to perform relevant calculations and evaluations of the study. The specific calculations of the cluster optimization algorithm are shown below.

The density peak-based clustering algorithm is to select cluster centroids based on *ρ*_*i*_ the measure of *δ*_*i*_ great local density and large distance and to divide the data by quickly searching for cluster centers and assigning noncluster center samples to the clusters where the nearest neighboring data points with greater local density than them are located [20]. The algorithm has two important metrics.

Local density, let *ρ*_*i*_ the dataset *D* = (*X*_1_, ⋯, *X*_*n*_) be for each data in *X*_*i*_ = (1, 2, 3, ⋯, *n*)*D* calculate its local density value, defined as

(1) $$\begin{array}{c} \rho_{i}=\underset{j}{\sum }e^{-dij/dc}. \end{array}$$

The distance between and high density *δ*_*i*_ points is the minimum value *i* of the Euclidean *ρ*_*i*_ distance between those points selected among all data points whose local *i* densities are larger than the data points, and the formula is shown in

(2) $$\begin{array}{c} \delta_{i}=\underset{j:\rho_{j}≻\rho_{i}}{\min}\left(d_{ij}\right), \end{array}$$

where *d*_*ij*_ is *i* the *j* Euclidean distance between the data and *d*_*c*_ is the truncation distance, in general, the distance between all data in ascending order after taking the first 1% to 2% of the distance as the truncation distance.

According to the above definition to calculate the corresponding value, *ρ* as the horizontal coordinates, as the vertical coordinates to generate a decision diagram, the determination of the cluster center requires a larger local *ρ*_*i*_ density and a larger and high-density *δ*_*i*_ point between the distance, that is, the cluster center is generally located in the upper right position of the decision diagram.

## 4. Results and Discussion

### 4.1. The Real Situation of Cultivating Labor Values among College Students in the New Era

“It is not easy to learn on paper, but it is necessary to do it by oneself.” In order to explore the problems of labor values of college students in the new era, this research conducted a questionnaire survey and carefully sorted them out in order to understand the current situation of the cultivation of labor values of contemporary college students through the actual survey and, on this basis, explore the reasons that hinder the progress of the cultivation of labor values and then provide some targeted strategies for the cultivation of labor values of college students. The answers to the above questions depend on the actual survey, so the conclusions of the article are based on the empirical research, mainly in the form of a questionnaire.

Having a correct knowledge of the connotation of labor lays a good foundation for the establishment of labor values. After the survey, it is found that college students at this stage can know the connotation of labor more correctly, but there is also a situation that they cannot understand labor in the new era accurately. In the survey on the connotation of labor, 46.92% of students think that labor is the activity of doing physical or mental work and creating material and spiritual wealth, 30.38% of students think that labor is the basis of social survival and development and a special form of human activity, and only 10.19% of students think that labor is the process of producing material materials, as shown in Figure 5.

In the understanding of the act of labor, according to the survey results, hard work, daily life labor, and internship, and practical training are all considered to be representatives of labor. This is shown in Figure 6.

In addition, 83.86% of the students think that there is no difference between high and low level of occupation, and no matter what kind of occupation they are going to engage in, as long as they work hard, they deserve respect. 68.65% of the students think that “labor is the most beautiful, glorious, great, and noble,” 33.85% of the students think that mental labor is better than physical labor, 21.92% of the students think that there is no need to promote the spirit of hard work in the new era, and 5.19% of the students think that housework is a matter for parents, so there is no need for children to interfere, as shown in Figure 7.

From this, it can be seen that most college students have a more correct perception of labor, but there are still a small number of students who do not have a clear and accurate perception of labor. The majority of college students can understand the connotation of labor more correctly and have a more accurate cognition of labor.

The majority of college students have a more accurate understanding of the value and choice of labor, and they can judge the role of labor in social development more correctly. In the new era, labor plays a very important role in social development, and the cognition of the role of labor can promote college students to make more correct value judgment. Regarding the value choice, on the one hand, take employment as an example. In response to the question of “what kind of job do you prefer after graduation?” In this question, most of the students prefer stable, interesting, and mental labor, and only 9.62% of them choose physical labor, which shows that most of the college students are still not willing to engage in physical labor. With the development of science and technology and the characteristics of the new era of college students, the type of labor represented by mental labor and stable labor has become the direction that the “00” college students pursue nowadays. Most of the students prefer second- and third-tier cities, their hometowns, and first-tier cities such as North, Shanghai, and Guangzhou, and only a small proportion of them choose remote areas such as Northwest China. The first choice, in addition, the main factors that affect the career choice of college students are welfare treatment, personal development space, whether the major is in line with personal interests, and the overall strength of the company, while social status has little influence on the new generation of college students, accounting for less than 20%. This shows that the new-age college students care more about the economic value brought by labor, which is a true reflection of the wealth value that labor can create, and they pay more attention to the future development, which shows that the new-age college students have their own clear plans for labor and pay less attention to the social status brought by labor to themselves. This is of great practical significance to their future development.

In addition, this paper also researches the development of the concept of “cultivating talents for the country” through the development of labor culture dissemination and ecological environment improvement. The study found that with the dissemination of labor culture and the improvement of ecological environment, the concept of “nurturing talent for the nation” has developed greatly, but the overall impact of the improvement of ecological environment on the concept is not as good as that of the dissemination of labor culture. This is shown in Figure 8.

### 4.2. Suggestions for Strengthening the Innovation of Labor Education in the New Era

How to make efforts in the innovation of labor education in colleges and universities and turn the tasks given by the times into practical actions, it is necessary to pay attention not only to the concept of strengthening the innovation of labor education but also to the majestic power brought by practical activities. Colleges and universities should face new problems and challenges, cooperate with multiple subjects to form a scientific value whole with internal and external linkage, so as to explore an effective path for innovation of labor education methods in colleges and universities in the new era.

1. Implement the spirit of innovation and enhance the innovative concept of colleges and universities. The innovation practice is led by the innovation concept, and whether the innovation concept is strong or not fundamentally determines the innovation effectiveness and even success or failure. To promote the innovation of talent development system and policy, colleges and universities should raise the banner of innovation of labor education method, focus on the central link of “educating talents for the country,” study and implement the spirit of innovation of labor education method as a whole, realize the idea first, let all teachers and students deeply experience the deep meaning of innovation of labor education method, and promote. The innovation of labor education method is internalized into spiritual pursuit and externalized into practical action

In-depth study of General Secretary Xi Jinping's important discourse on innovation, through teacher training, thematic report meetings, and thematic class meetings, we will study the spirit and rich connotation of the innovation of labor education methods in the new era in depth and implant the innovation of labor education methods deeply into our minds so that teachers know how to innovate and have the ability to innovate. To enhance students' innovative ideas, we can carry out labor education-themed entrance education activities during the new students' entrance stage, convey the spirit and stories of model workers to students, and invite outstanding labor representatives of our school to tell the deeds of model workers at the training site so that students feel more intimate and the education effect is more obvious. Be a good advocate of the concept of innovation in labor education methods, pay attention to establishing the concept of innovation in labor education methods among teachers and students, and guarantee the efficient promotion of innovation in labor education methods.

(2) To carry out thematic training, teachers are the practitioners of the innovation of labor education methods, and a correct understanding of the innovation of labor education methods is an important prerequisite. If teachers do not have a deep enough understanding of the labor education approach, they are bound to operate deformation in the practice of labor education approach innovation. To achieve innovation in labor education methods in this context, it is necessary to change teachers' cognition of innovation in labor education methods. Colleges and universities should strengthen teachers' professional training to enhance their cognition of labor education approach innovation. Motivate teachers to be active in the innovation of labor education methods and take the initiative to contribute their own strength to the innovation of labor education methods
(3) Promote the awareness of innovation and strengthen students' innovative ideas. In the new era, China is in the stage of high-quality development, and the country needs talents with innovative ideas to achieve innovative development and should pay attention to the innovation of labor education methods. Students in the new era should focus on solving problems that cannot be solved by existing methods and approaches, always with a sense of worry and innovation, and also focus on solving and preventing new problems and challenges to be faced in the future, combining the spirit of innovation with the attitude of seeking knowledge and enhancing the confidence, courage, and ability to cultivate innovation

#### 4.2.1. Keeping in Mind the Original Intention of Nurturing Talents for the Country, Strengthen the Sense of Innovation in Labor Education Methods

In recent years, the development of colleges and universities also puts innovation in the core position, deeply explores the advantages of using resources, makes efforts to strengthen the construction of innovative colleges and universities, and promotes the national innovation-driven development to achieve new breakthroughs. It is deeply aware of the changes in the innovation environment of labor education methods, further optimizing the innovation environment of labor education methods, enhancing the innovation consciousness of labor education methods, and accelerating the pace of construction of innovative universities.

Implement the spirit of innovation and enhance the innovative concept of colleges and universities. The concept is the precursor of action, and the innovation practice is led by the innovation concept, and whether the innovation concept is strong or not fundamentally determines the innovation effectiveness and even success or failure. To promote the innovation of talent development system and policy, colleges and universities should raise the banner of innovation of labor education method, focus on the central link of “educating talents for the country,” study and implement the spirit of innovation of labor education method as a whole, realize the idea first, let all teachers and students deeply experience the deep meaning of innovation of labor education method, and promote. The training will help teachers and students deeply appreciate the deeper meaning of the innovation of labor education methods and promote the innovation of labor education methods to be internalized into spiritual pursuit and externalized into practical action.

To carry out thematic training, teachers are the practitioners of labor education innovation, and a correct understanding of labor education innovation is an important prerequisite. If teachers do not have a deep enough understanding of labor education methods, they will definitely operate deformation in the practice of labor education method innovation. In this context, in order to realize the innovation of labor education method, it is necessary to change teachers' cognition about the innovation of labor education method. Higher education institutions should strengthen teachers' professional training to enhance their cognition of labor education approach innovation.

Propagate the awareness of innovation and strengthen students' innovative ideas. Strengthen the concept of innovation, expand scientific knowledge, and promote the unity of knowledge and action. College students' minds are not yet mature enough to use scientific theories to discriminate when facing the intrusion of undesirable external trends in order to avoid themselves from falling into the whirlpool of finalization and secularization. Continuously optimize the way and method of learning, improve the consciousness of learning, and enhance cultural self-confidence. Adhere to the practice of linking theory with practice, actively learn to master scientific and cultural knowledge, use the deeds of model workers to inspire themselves, use the power of role models to spur themselves on, use excellent traditional culture to inculcate themselves, learn from the advanced to love their jobs and strive for first-class dedication, and lay down the fundamental guarantee of establishing themselves and building the foundation of serving the country.

#### 4.2.2. Establish and Improve Institutional Mechanisms to Stimulate the Innovation of Labor Education Methods

1. Form a guarantee mechanism to ensure innovation conditions. The innovation of labor education methods in colleges and universities depends on the leadership of innovative ideas and scientific and reasonable evaluation system. At the same time, it also needs the support and guarantee of conditions in all aspects. Organizational attention, reasonable staffing mechanism, financial investment, and sufficient practice sites are all necessary to ensure the innovation of labor education methods

Scientific organization and implementation mechanism of labor education, according to the requirements of the documents about strengthening labor education, colleges and universities seriously implement the spirit of the documents and include the innovation of labor education methods in the labor education plan, taking into account the actual local conditions. The leaders of colleges and universities should establish a sound labor education organization and implementation work mechanism, clarify the hierarchical supervisors, and specify the responsibilities of each department to guarantee the orderly development of labor education. For example, Zhengzhou Shengda College of Economics, Trade, and Management makes clear the leaders in charge in the labor education implementation system, establishes a labor education management organization—Labor and Health Section, and also has two full-time personnel to supervise and oversee the implementation of labor education so that the implementation is carried out at all levels and responsibilities are assigned to people, which effectively improves the problem of vapid labor education way innovation.

(2) Writing the effect of labor education into the evaluation index of colleges and universities to improve the motivation of innovation of labor education methods in colleges and universities, quality assessment of higher education is a concern of college reform. Although higher education teaching assessment has effectively promoted high-quality development of higher education institutions, it also presents many problems. For example, the subjects of assessment are not diversified and scientific enough, and colleges and universities perform passively. In order to stimulate the independent creativity and initiative of colleges and universities, they should be encouraged to combine the advantages of our university and build unique and attractive colleges and universities. Let colleges and universities get comprehensive, active, and sustainable development and stimulate the independent innovation ability of colleges and universities. The government should also take the initiative to give policy support and pay attention to the educational function of assessment. The phenomenon of vain and weak innovation of labor education methods in colleges and universities is largely due to the fact that the leaders of colleges and universities do not pay enough attention to the innovation of labor education methods. Therefore, the effect of labor education can be included in the important indexes of higher education evaluation, so as to stimulate the enthusiasm of labor education method innovation
(3) The objectives of evaluation should be in line with reality. Colleges and universities should fully grasp the law of college student development and the law of education development, clarify the development stage and environment in which the university is located, and combine their own development plans and goals. The form of assessment should be diversified, reflecting quantitative and taking into account qualitative, adding self-assessment and other assessment. In a fixed period of time, an evaluation team composed of teachers, students, and expert teachers is set up to give a comprehensive evaluation of the implementation of labor education for students. This kind of evaluation can provide visual feedback on the effect of labor education and facilitate the labor education guidance department to update the indicators of evaluation in time

#### 4.2.3. Deepen Offline-Online Integration and Broaden the Innovative Platform of Labor Education Methods

The diversification of labor education contents determines the diversification of labor education methods. With the development of the times and the progress of information technology, the content of labor education has become more colorful, and “online learning” has become the learning method of many students. This also determines that the innovation of labor education methods should be made in the direction of integrating online and offline and broadening the platform for innovation of labor education methods.

Integrating labor education courses into on-campus labor practices, there are many real labor practice opportunities on campus. The content of labor education courses can be combined with dormitory hygiene cleaning, logistics work, cafeteria work, campus greening, and also with assistant supervisors, assistant teachers, on-campus tour guides, and exhibition lectures to provide students with labor practice opportunities and enrich the content and methods of labor education courses. Adhere to the orientation of nurturing people and always take cultivating the new man of the times as the goal of education. Grasp the value orientation of labor education, fully respect the characteristics of students' subjects, guide students' love for labor, advocate the democratization of the choice of labor education methods, and fully mobilize students' enthusiasm. In order to improve the attractiveness of labor education courses and enrich labor education methods, Zhejiang Agriculture and Forestry University has opened four labor education on-campus practice courses, including learning to cook fish with a famous chef, planting trees and flowers with a green master, and learning storage with a host teacher. Henan University of Technology explored a new model of labor+education, playing the role of school logistics, online “basic maintenance of life,” “dormitory life experience,” and other labor education “new classroom.”

The labor education courses are conducted online and offline with the full use of integrated media resources. With the development of science and technology, education and teaching are also being reformed. Modern network technology has played a good role in education, and the teaching content has been integrated with intelligent elements so that students can enjoy colorful teaching content. Course theory teaching has been as an important form of teaching. Therefore, colleges and universities should actively use network resources, use intelligent technology, and innovate labor education methods. By combining with network resources, the classroom does not have the boundary of inside and outside the school. The innovative curriculum approach will improve the labor education approach system and fully realize the important function of curriculum education.

## 5. Conclusion

The innovation of labor education methods in colleges and universities is crucial. In the new era, colleges and universities cultivate knowledge-based, technical, and innovative talents with comprehensive development, which can effectively enhance the core competitiveness of college students in employment. Labor education plays an important role in the goal of comprehensive development education, and it is reasonable to conduct systematic research on the innovation of labor education methods in colleges and universities to enhance the effectiveness of labor education in colleges and universities and accelerate the realization of the Chinese dream of great innovation of the Chinese nation. Through the research on the innovation of labor education methods in colleges and universities in the new era, the core connotation and value implication of the innovation of labor education methods in colleges and universities in the new era are deeply understood. Based on the broad perspective of integrating theory and reality, General Secretary Xi Jinping pointed out the historical responsibility and mission of the times that colleges and universities shouldered and gave the target orientation and basic direction for the innovation of labor education methods in colleges and universities in the new era. The effect of innovation of labor education methods in colleges and universities maps the development direction of future society. Although the overall innovation of labor education methods in colleges and universities is good, there are still phenomena of deficiency, weakness, simplicity, and fragmentation. The reasons for the problems of labor education innovation in colleges and universities include five aspects: the innovation of labor education in colleges and universities emphasizes general propaganda, light on specific practice and continuity of inheritance, innovation of revolution and imitation, originality of characteristics and rich content, development of carrier, local breakthrough, and overall promotion. On this basis, colleges and universities should bear in mind the original intention of educating talents for the country and enhance the awareness of innovation of labor education methods among teachers and students. The innovation of labor education methods should be emphasized in the preservice and postservice training of teachers, and the innovation of labor education methods should be promoted in the entrance training and daily class meetings of students. In order to stimulate the vitality of labor education method innovation in colleges and universities, colleges and universities should form guarantee mechanism, formulate incentive mechanism, standardize evaluation system, promote curriculum integration, broaden practice channels, and tap network resources as a way to broaden the platform of labor education method innovation. In cooperation with families, schools, and society, we should strengthen the communication between them and join hands with each other to optimize the environment of labor education innovation. In the new era, the innovation of labor education in colleges and universities faces great opportunities, and the strategic development goal of China's innovation provides a superior environment for the development of innovation of labor education.

## Figures and Tables

**Figure 1:** Theoretical significance of labor education.

**Figure 2:** The five-education and three-whole philosophy.

**Figure 3:** Habitat focus areas of work.

**Figure 4:** History of the development of ecological and environmental theory.

**Figure 5:** Understanding of the connotation of labor.

**Figure 6:** Understanding of labor behavior.

**Figure 7:** Understanding of the connotation of labor in the new era.

**Figure 8:** The influence of labor culture dissemination and ecological environment improvement on the concept of “cultivating talents for the nation.”

## Data Availability

The labeled dataset used to support the findings of this study is available from the corresponding author upon request.
